The article "Traditional Chinese Medicine Formula Jian Pi Tiao Gan Yin Reduces Obesity in Mice by Modulating the Gut Microbiota and Fecal Metabolism" was published in 2022. Journal: Evid Based Complement Alternat Med.

# Traditional Chinese Medicine Formula Jian Pi Tiao Gan Yin Reduces Obesity in Mice by Modulating the Gut Microbiota and Fecal Metabolism

**DOI:** 10.1155/2022/9727889

**Published:** 2022-08-08

**Authors:** Wenchao Dong, Yulin Mao, Zhenhua Xiang, Jingyu Zhu, Haixia Wang, Aiju Wang, Meifang Jiang, Yuming Gu

**Affiliations:** ^1^Department of Traditional Chinese Medicine, Affiliated Hospital of Weifang Medical University, School of Clinical Medicine, Weifang Medical University, Weifang 261042, China; ^2^Weifang Medical University, Weifang 261042, China; ^3^Clinical Research Center, Affiliated Hospital of Weifang Medical University, Weifang 261042, China

## Abstract

The current study employed the high-fat diet (HFD) induced murine model to assess the relationship between the effect of Jian Pi Tiao Gan Yin (JPTGY) and the alterations of gut microbiota and fecal metabolism. C57BL/6 mice were used to establish an animal model of obesity via HFD induce. Serum biochemical indicators of lipid metabolism were used to evaluate the pharmacodynamics of JPTGY in obese mice. Bacterial communities and metabolites in the feces specimens from the controls, the Group HFD, and the JPTGY-exposed corpulency group were studied by 16s rDNA genetic sequence in combination with liquid chromatography-mass spectrometry (LC-MS) based untargeted fecal metabolomics techniques. Results revealed that JPTGY significantly decreased the levels of total cholesterol (TC), triglyceride (TG), low-density lipoprotein cholesterol (LDL-C), and elevated high-density lipoprotein cholesterol (HDL-C). Moreover, JPTGY could up-regulate the abundance and diversity of fecal microbiota, which was characterized by the higher phylum of proteobacteria. Consistently, at the genus levels, JPTGY supplementation induced enrichments in *Lachnospiraceae NK4A136 group*, *Oscillibacter*, *Turicibacter*, *Clostridium sensu stricto 1*, and *Intestinimonas*, which were intimately related to 14 pivotal fecal metabolins in respond to JPTGY therapy were determined. What is more, metabolomics further analyses show that the therapeutic effect of JPTGY for obesity involves linoleic acid (LA) metabolism paths, alpha-linolenic acid (ALA) metabolism paths, glycerophospholipid metabolism paths, arachidonic acid (AA) metabolism paths, and pyrimidine metabolism paths, which implied the potential mechanism of JPTGY in treating obesity. It was concluded that the linking of corpulency phenotypes with intestinal flora and fecal metabolins unveils the latent causal link of JPTGY in the treatment of hyperlipidemia and obesity.

## 1. Introduction

According to the latest data, more than 1.9 billion adults across the globe are overweight and over 600 million are obese [1]. Corpulency has become a global epidemic [2]. Obesity is not only a potential condition for chronic inflammatory and metabolic diseases [3] but also obesity-related cardiovascular illnesses, type 2 diabetes mellitus (T2DM), nonalcoholic fatty liver illness, and other diseases have become major challenges to global health [4].

The intestinal flora participates in modulating the completeness of the intestine mucosa barrier, nutrient absorption, and fat metabolism and storage [5–8]. Several pieces of research have shown that the intestinal flora has a complex relationship with the occurrence and progression of corpulency, and is also associated with other metabolism illnesses in obese patients such as hypertension, diabetes, cardiovascular disease, and chronic kidney disease [9]. The intestinal flora enriched in the cecum and colon can metabolize dietary fiber, protein, polypeptides, and other substances that are hard to digested by host enzymes, and the specific genus or different abundance of bacteria has a certain impact on obesity and other metabolic diseases [10]. It has already been revealed that germ-free mice colonized with an “obese microbiome” have increased energy absorption and total body fat [11]. The intestinal flora exerted a vital regulatory effect on obesity pathophysiology and related diseases through the regulation of intestinal appetite-stimulating hormone, changes in insulin resistance (IR), nutrient digestion, energy regulation, glucose metabolism, and lipid metabolism [1, 11–13]. Therefore, more and more studies are also focusing on intestinal microflora as a latent treatment target to avoid and improve obesity and its related metabolic diseases.

Metabolomics aims to study the metabolic changes of low molecular weight endogenous and exogenous metabolites in the biological system through modern analytical techniques and has huge advantages for the research of complex systems, such as studies of metabolic diseases and the mechanisms of traditional Chinese medicine (TCM) [14–16]. The non-targeted metabolomics is predominantly utilized to identify markers and investigate causal links via the search for differential metabolins between experiment and control groups along with the analysis of metabolism paths, hence, it is extensively utilized to research metabolism-related illnesses [17]. The cumulation of proofs related to metabolism variations is vital for facilitating TCM therapies to treat corpulency.

In recent years, the interplay between obesity, intestinal flora, and Chinese herbal medicine has attracted widespread attention. Obesity-induced by long-term consumption of HFD can cause significant changes in intestinal microbes and metabolites [18]. Mounting evidence has demonstrated that TCM can modulate the body's metabolic process via the gut microbiome and its metabolins, and can realize treatment effects in corpulent individuals [19–22]. Chinese herbal medicines have been shown to regulate the composition of intestinal flora, fecal short-chain fatty acids (SCFAs), intestine barrier functions, and intestinal inflammatory events [23].

Jian Pi Tiao Gan Yin (JPTGY) is an effective prescription for obesity treatment based on our long-term clinical practice. It is effective in soothing the liver, regulating qi, strengthening the spleen, and resolving phlegm. In the earlier period, our group found that JPTGY has a satisfactory effect on weight loss in patients with obesity. JPTGY has markedly reduced total cholesterol and triglyceride levels in patients, without any side effects [24]. The JPTGY decoction was constituted by *Astragalus* (Sheng Huang Qi), Bupleurum (Chai Hu), Poria cocos (Fu Ling), Salvia miltiorrhiza (Dan Shen), Coix seed (Yi Ren), Radix Paeoniae Alba (Bai Shao), Cassia seed (Jue Ming Zi), Herba eupatorii (Pei Lan), Rhizoma alismatis (Ze Xie), Rheum officinale Baill (Shu Da Huang), and Hawthorn (Shan Zha). Our animal experiments have confirmed that JPTGY has a significant weight loss effect on corpulency caused by HFD in rats and mice [25]. JPTGY also can increase the expressions of *UCP-1* and *PGC-1α* mRNA in adipose tissue of mice [26]. These studies indicated that the mechanism of JPTGY in treating obesity involves elevation of the browning of white adipose and regulation of intestinal flora, which suggests that JPTGY was a promising compound with good drug ability. Nevertheless, due to the characteristics of traditional Chinese medicine formulation being multi-way and multi-target, the mechanism of JPTGY in treating obesity is not sufficient.

Therefore, the present research intended to detect the regulatory role of JPTGY in intestinal microflora and metabolites of obese mice by 16S rDNA sequencing technology and LC/-MS non-targeted fecal metabolomics studies, further unveiling the underlying mechanism of action for the lipid-lowering effect of JPTGY and its possible role in reducing weight in HFD mice.

## 2. Materials and Methods

### 2.1. Preparation of Jian Pi Tiao Gan Yin

The TCM formula herein was JPTGY, comprising 11 herbal medicines: Astragalus (Sheng Huang Qi), Bupleurum (Chai Hu), Poria cocos (Fu Ling), Salvia miltiorrhiza (Dan Shen), Coix seed (Yi Ren), Radix Paeoniae Alba (Bai Shao), Cassia seed (Jue Ming Zi), Herba eupatorii (Pei Lan), Rhizoma alismatis (Ze Xie), Rheum officinale Baill (Shu Da Huang), and Hawthorn (Shan Zha).Herbal medicines were offered and their qualities were supervised by our hospital (PRC). Details are as follows: The entire herbal medicines were boiled for two times, 600 s with high heat and afterward 20 min with gentle heat posterior to the 0.5-h soaking. The decoction was subjected to filtration with 2-tier gauze to discard remains and then heated to 2.00 g/ml, and finally, it was preserved under 4°C.

### 2.2. Animals and Experiment Design

Five-week-old male C57BL/6J mice (*n* = 30) were provided by the Medical Laboratory Animal Center of Weifang Medical University and were housed at 23 ± 2°C and a comparative humidity of 50 ± 10% with a 12-h light/dark period. All of the animal assays were performed at the Medical Laboratory Animal Center of Weifang Medical University. The Guidance for Lab Animal Welfare and Utilization was followed [27]. After 7 days of acclimatization, mice were separated into 3 groups: (1) the Group NC (*n* = 10), fed a normal chow diet (1010009 diets, 12.79 kcal% fat, Jiangsu Synergy Medicine Bioengineering Co., Ltd.); (2) the Group HFD (*n* = 10), fed an HFD (XTHF60-1 diet, 60.65 kcal% fat, Jiangsu Synergy Medicine Bioengineering Co., Ltd.); and (3) the Group JPTGY (*n* = 10), HFD supplied with JPTGY. The Group JPTGY has gavaged 6 ml of 12 g/kg. BW JPTGY oral liquid intragastric administration, while mice in Group NC and Group HFD received 6 mL of distilled water intragastric administration. Gavage was given twice a day at 8∶00 and 16∶00 separately for 12 successive weeks. The body weight of mice and food consumption were identified every week. At the end of the assay, animals were fasted for 4 h prior to the retro-orbital blood withdrawal. Subsequently, feces specimens were collected for analysis. To be specific, intestinal feces were collected and preserved under −80°C for 16S rDNA genetic sequence identification and LC-MS-based untargeted fecal metabolomics studies.

### 2.3. Biochemical Analysis

Blood specimens were kept still for 120 min prior to the centrifugation at 3000 rpm for 15 min under 4°C. Subsequently, supernate was extracted for blood biochemical assay. Serum levels of TC, TG, HDL-C, and LDL-C were identified via the assay kits (Changchun Huili Biological Technology Co., Ltd. China).

### 2.4. Gut Flora Sequencing and Data Analyses

Partial feces specimens were sent to the Shanghai Lu-Ming Biotechnology Company (PRC, https://www.lumingbio.com) for 16S rDNA genetic sequence identification. Overall genome DNA was abstracted via a DNA extraction tool as per the supplier's specification. The content of DNA was validated via NanoDrop and agarose gel. For microbial diversity analyses, V3–V4 variable areas of 16S rRNA genes were magnified via universal primers 343 F and 798 R. Raw sequence identification information were in FASTQ format. Paired-end reads were afterward preprocessed via Trimmomatic program [28] to identify and cut off ambiguous bases (N). It also discarded low-quality results with mean quality scoring ＜ 20 via the sliding window trimming method. Subsequently, paired-end reads were assembled via the FLASH program [29]. The assembly variables were: 10 bp of minimum superimposition, 200 bp of maximal superimposition, and 20% of maximal mismatch rate. The denoising was completed via: reads with ambiguous, homologous sequences or below 200 bp were discarded. Reads with 75% of bases above Q20 were kept. Afterward, reads with chimera were identified and discarded. Those 2 steps were completed via the QIIME program [30] (v 1.8.0). Clean reads were treated with primer sequence removal and clustering to produce operational taxonomic units (OTUs) via the VSEARCH program [31] with 97% resemblance cutoff. The typical read of every OTU was chosen via the QIIME package. Every typical read was annotated and blasted against Silva database v123 via the RDP classifier [32] (confidence liminal value was 70%).

Five samples were randomly selected from each group for analysis. The richness, Shannon diversity, Chao1, phylogenetic diversity indices, as well as rarefaction curves were computed via QIIME (v 1.9.1) and demonstrated via R program (v 3.2.2). The alpha diversity was utilized Wilcoxon rank-sum test for comparing statistically significant diversities amongst groups. For bacterial community analysis (each group, *n* = 5), nonmetric multidimensional scaling (NMDS) was demonstrated via a vegan package in R program (v 3.2.2). Remarkable diversities in phylum levels and F/B ratio between 2 groups were computed via R program for *t*-test to acquire *p* results. Linear discriminant analysis (LDA) effect size (LEfSe) in combination with the normal tests (Kruskal–Wallis rank-sum test and Wilcoxon rank-sum test) with LDA was utilized for comparing statistically significant diversities, and the *α*-value was fixed to <0.05, and the threshold used to consider a discriminative feature for the logarithmic LDA score was set to >3.0. The functional potential of the bacterial community based on 16S rDNA gene sequencing was predicted by using PICRUSt2.

### 2.5. LC/MS Nontargeted Metabolomics Study and Data Analysis

Partial feces specimens were sent to Shanghai Lu-Ming Biotechnology Company (PRC, https://www.lumingbio.com) for LC/MS non-targeted metabolomics study.

A fecal sample (30 mg) was weighted to an EP tube, and a 400 *μ*L extract solution (methanol: water = 4 : 1) was added. Then they were homogenized by a JXFSTPRP-24/32 automatic sample fast grinder for 2 min at 60 Hz. Next, they were vortexed for half a minute and ultrasonicated for 10 min at 40 kHz (incubated in ice water). The mixture was incubated for 30 minutes at −20°C to precipitate proteins and then centrifuged at 13,000 rpm for 10 min at 4°C. The supernate (150 *μ*L) from all tubes was harvested via crystal syringes, subjected to filtration via 0.22 *μ*m microfilters, and moved to LC phials. Phials were preserved under −80°C for LC-MS analyses.

An ultra performance liquid chromatography system (ThermoFisher, China) was applied to achieve chromatographic separations. Reversed-phase separation was performed on an ACQUITY UPLC HSS T3 column (100 mm × 2.1 mm, 1.8 *μ*m). The temperature was set at 45°C, the flow rate was 0.35 mL/min, and the injection volume was 2 *μ*L. The mobile phase was composed of solvent A (water, 0.1% formic acid) and solvent B (acetonitrile, 0.1% formic acid). Gradient elution parameters were set as follows: 0.01∼2 min, 5% B; 2∼14 min, 5% to 100% B; 14∼15 min, 100% B; 15∼15.1 min, 100% to 5% B; and 15.1∼18 min, 5% B.

Metabolites were detected by high-resolution tandem mass spectrometer QE (ThermoFisher, China) in both negative and positive ion models. The mass range was between m/*z* 100 and 1000. The resolution was 70,000 for the full MS resolution and 1,7500 for MS/MS resolution. The Collision energy was 10, 20, and 40 eV. The mass spectrometry detector was run as follows: spray voltage, 3,800 V (+) and 3,200 V (−); sheath gas flow rate, 40 arbitrary units; auxiliary gas flow rate, 8 arbitrary units; and capillary temperature, 320°C. The QCs were introduced via injection regularly (every 10 specimens) across the analytic run to offer data from that repetitiveness can be evaluated.

Non-targeted liquid chromatography-mass spectrometry (LC-MS) analyses were performed for peak detection and comparison by importing the raw data into the Progenesis QI 2.3 software program (Nonlinear Dynamics, Newcastle, UK), and a data matrix composed of retention time (RT), peak intensity and mass-to-charge ratio (m/*z*) values were obtained. Additionally, qualitative and quantitative information for specific metabolites was acquired. Preprocessing was necessary before the multivariate statistical analysis, and the methods were as follows: (1) data were removed if missing values contained more than 50% in the sample; (2) based on one-half of the minimum metabolite value, the missing values were filled and the total peaks were normalized; and (3) QC samples were eliminated if the relative standard deviation (RSD) was more than 30%. Finally, logarithmic transformation was performed for preprocessed datasets prior to further analysis. Mass spectra of these metabolic features were identified by using the accurate mass, MS/MS fragments spectra, and isotope ratio difference by searching in reliable biochemical databases, such as Human Metabolome Database (HMDB) and Kyoto Encyclopedia of Genes and Genomes (KEGG). Specifically, the precursor tolerance was 5 ppm/10 ppm, product tolerance was 10 ppm/20 ppm. For MS/MS-confirmed metabolites, only metabolites with MS/MS fragment scores abovementioned 36 were considered reliably and identified. Otherwise, the metabolites had only tentative assignments.

Seven fecal samples were randomly selected from each group for analysis. For metabolomic data (each group, *n* = 7), partial least-squares-discriminant analysis PLS-DA was performed for visualizing the metabolism variations among different condition groups, posterior to mean log transformation and auto-scaling, separately. To identify the most vital variations in diverse circumstances, the volcanic plot was utilized to find the differential metabolites. The bacteria-metabolin association was assessed by a heat map produced from the computation of the Pearson correlation coefficient for every pairwise combination of microbe genus richness and metabolin intensity via the “CORR-test” function in the “psych” *R* package. In addition, the differential metabolites were processed and studied by Metabo Analyst 5.0, via the pathway analyses module (https://www.metaboanalyst.ca/MetaboAnalyst/). Wilcoxon rank-sum test was used to identify biochemicals that differed significantly between the two groups.

### 2.6. Statistical Analysis

The data were displayed as average ± SD. Statistically significant diversities were evaluated via the one-way ANOVA by GraphPad Prism 9.0 software. For metabolomic data, Wilcoxon rank-sum test was used to identify biochemicals that differed significantly between the two groups. *p* values were corrected for multiple comparisons using the Benjamini–Hochberg false discovery rate (FDR) control procedure, and *p* < 0.05 had significance on statistics in this work.

## 3. Results

### 3.1. JPTGY Attenuated Hyperlipidemia in HFD-Fed Mice

At the end of the experiment, our team detected lipid levels (TC, TG, HDL-C, and LDL-C) for each mouse. As indicated in Figure 1, the rats fed HFD remarkably elevated the TC, TG, and LDL-C contents and reduced the serum HDL-C content (*p* < 0.05), in contrast to NC mice. Moreover, with JPTGY treatment, the serum TC, TG, and LDL-C contents of HFD rats were remarkably decreased vs. HFD mice (*p* < 0.05). In addition, serum HDL-C contents of the Group JPTGY had increased vs. HFD mice (*p* < 0.05). The outcomes herein revealed the JPTGY treatment could mitigate the hyperlipoidemia caused by HFD.

### 3.2. JPTGY Regulated the Overall Structure of the Intestinal Flora in HFD-Induced Obese Mice

For the sake of examining the roles of HFD and JPTGY in the intestinal flora, the rarefaction curve has attained a steady status, which revealed that the sequence identification has covered rare new phenotypes and satisfied the most diversities (Figure 2).

Alpha diversity analysis denotes the diversity and richness of species in the biological environment. It is well known that obese individuals usually show reduced diversity and richness of intestinal bacteria [33]. In our study, a significantly reduced index of richness was found in the Group HFD compared with the Group NC (*p* < 0.05, Figure 3(a)). In contrast to HFD, JPTGY mice had elevated index for the entire 4 variables, among which the variations in abundance displayed significance on statistics (*p* < 0.05, Figure 3(a)). Notably, a significantly increased index of Chao1 and phylogenetic diversity was found in the HFD mice vs. the NC mice (*p* < 0.05, Figures 3(c) and 3(d)). This may be due to the small number of rats, or to the fact that the composition of gut microbes is related to the quality and quantity of fat in high-fat diets [34]. WANG B et al. also proposed that the increase of fiber content in HFD might be the reason for the increased diversity of intestinal flora in the Group HFD [35]. In general, our result suggested that JPTGY elevated intestinal flora diversity and richness in the HFD mice. Venn diagram analysis provides a better understanding of bacterial abundance in all groups (Figure 3(e)). The results showed that 2362 cases of OTU overlapped in each group. There were 266 OTUS specific in the Group NC, 191 OTUS in the Group HFD, and 171 OTUS in the Group JPTGY. To further understand the effects of HFD and JPTGY on the architectures and constituents of gut microbiota, beta diversity analysis, and sample tree clustering were performed. It can be seen that there were different collections in the three groups, indicating that the separation degree among the groups was good, and there were certain differences in intestinal microbial structure (*p* < 0.05, Figure 4(a)). Moreover, in the sample tree clustering analysis (Figure 4(b)), we found that Group HFD was closer to Group NC, while Group JPTGY was far away from Group NC. Beta diversity analysis showed that diet played a key role in the formation of intestinal microflora. Different dietary treatments (NC, HFD, and JPTGY) produced different intestinal microflora, and JPTGY could significantly regulate the composition of intestinal microflora in HFD mice.

### 3.3. JPTGY Modulated Intestinal Flora at Phylum Levels in HFD Mice

At the phylum level, the top 10 phyla in the relative richness of intestinal flora were displayed as histograms (Figure 5(a)), where *Firmicutes* and *Bacteroidetes* were listed as the top 2 predominant phyla in every group, accounting for more than 90% of the total phyla in the three groups. Furthermore, contrast revealed that relative to NC mice, HFD mice had remarkably elevated the relative richness of *Firmicutes* and *Proteobacteria*, but decreased the relative richness of *Bacteroidetes*. However, JPTGY-exposed animals displayed no remarkable effects on the relative richness of *Firmicutes* and *Bacteroidetes* (*p* > 0.05, Figure 5(a)), but remarkably decreased the relative richness of *Proteobacteria* (*p* < 0.05, Figure 5(a)). Moreover, our team contrasted the ratio of F/B as a sign of corpulency amongst these 3 groups. As presented in Figure 5(b), HFD remarkably elevated the ratio of F/B *p* < 0.05), its effect could be terminated by JPTGY but no remarkable diversities existed between HFD mice and JTPGY (*p* > 0.05).

### 3.4. The Dominant Microbiota among Different Treatment Groups

The LEfSe analysis further explored the dominant microbiota (taxa with remarkably diverse richness and effects, LDA >3) amongst diverse therapy groups. The outcomes in Figures 6(a) and 6(b) revealed that *Bacteroidales*, *Bacteroidia*, *Bacteroidetes*, *uncultured bacterium*, *Muribaculaceae*, *Unsigned*, *uncultured Bacteroidales bacterium*, *Alistipes*, *Rikenellaceae*, and *Muribaculum* were predominant microbes community in NC mice. The dominant bacteria in Group HFD were *Firmicutes*, *Clostridia*, *Clostridiales*, *Lachnospiraceae*, *uncultured_organism*, *Ruminococcaceae*, *Lachnoclostridium*, *Ruminococcaceae UCG 014*, *Ruminiclostridium*, *Bacilli*, *Lactobacillales*, *Lactobacillaceae*, *Lactobacillus*, *Lachnospiraceae UCG 006*, *Proteobacteria*, *Actinobacteria*, *Coriobacteriales*, *Coriobacteriia*, *Eubacterium xylanophilum group*, *Atopobiaceae*, *Lachnospiraceae UCG 001*, *Coriobacteriaceae UCG 002*, *Desulfovibrio*, *Desulfovibrionaceae*, *Desulfovibrionales*, and *Blautia*. JPTGY supplementation induced enrichments in *Lachnospiraceae NK4A136 group*, *Oscillibacter*, *Turicibacter*, *Clostridium sensu stricto 1*, *Clostridiaceae 1*, *Erysipelotrichia*, *Erysipelotrichales*, *Erysipelotrichaceae*, *Parvibacter*, *gut_metagenome*, and *Intestinimonas*. A cladogram displaying the taxonomical hierarchic architecture of the feces flora from phylum to species revealed remarkable diversities in phylogenesis distribution among the microbial communities of NC mice, HFD mice, and JPTGY mice (Figure 6(b)). Those outcomes revealed an evident diversity in feces flora constituents between the Group NC, HFD, and JPTGY. In addition, *Actinobacteria* were found to be particularly enriched in HFD while it played unfavorable roles in obesity prevention.

### 3.5. Functional Prediction of Intestinal Flora in PICRUSt2

According to the KEGG database, PICRUSt2 analyses on the foundation of 16S rDNA genetic sequencing information were utilized to study the intestinal flora function associated with JPTGY therapy. As shown in Figure 7, lipometabolism, energy metabolic process, glycan synthesis and metabolic process, transportation and katabolism, metabolic process of terpenoids and polyketides, carbohydrate metabolic process, nucleotide metabolic process, and amino acid metabolic process were up-regulated in Group JPTGY.

## 4. Results of Fecal Metabolomics Analysis

Our team completed global metabolomics profiling analyses via lyophilized feces specimens to observe the metabolism status of NC, HFD, and JPTGY mice. The PLS-DA score plot showed a significant separation effect between samples of Group NC, HFD, and JPTGY (Figure 8(a)). In our study, for the sake of identifying the most vital variations in diverse circumstances, we used volcanic plots to find the differential metabolites (Figures 8(b)–8(d)). The results showed a total of 20 enriched metabolites involved in metabolism in Group HFD and JPTGY (Figure 8(e)).

As described above, the LEfSe analysis indicated that Group HFD-induced enrichments in *Ruminococcaceae UCG 014*, *Ruminiclostridium, Lactobacillus*, *Lachnospiraceae UCG 006*, *Lachnospiraceae UCG 001*, *Lachnoclostridium*, *Eubacterium xylanophilum group*, *Desulfovibrio*, *Coriobacteriaceae UCG 002*, and *Blautia* at the genus level. And the JPTGY supplementation induced enrichments in *Turicibacter*, *Oscillibacter*, *Lachnospiraceae NK4A136 group*, *Intestinimonas*, and *Clostridium sensu stricto 1* at the genus level. In this regard, we performed Pearson correlation analysis between the predominant microbes at the genus level and the 20 enriched fecal metabolites.

The heatmap in Figure 8(e) displayed those 15 enrichment genera were positively or negatively related to the 20 enriched fecal metabolites, which belonging phenols, fatty acyls, glycerophospholipids, prenol lipids, sphingolipids, carboxylic acids and derivatives, indoles and derivatives, imidazopyrimidines, stilbenes, and stilbenes. It was revealed that *Turicibacter* enriching in Group JPTGY was significantly positively correlated to the C17 sphingosine-1-phosphocholine (*p* < 0.05). Moreover, the metabolites levels of the 2-O-(beta-D-galactopyranosyl-(1->6)-beta-D-galactopyranosyl) 2S-hydroxynonanoic acid, 2-((1Z)-1-(4-(2-(dimethylamino) ethoxy)phenyl)-2-phenyl but-1-en-1-yl)phenol and dolasetron were significantly negatively correlated with the abundance of *Oscillibacter* enriching in Group JPTGY, but significantly positively correlated with the *Lactobacillus* enriching in Group HFD (*p* < 0.05). *Lachnospiraceae UCG 006*, *Lachnoclostridium*, and *Blautia*enriching in Group HFD were significantly positively correlated to S-japonin while (1(10)E,4E,6a,8b)-8-angeloyloxy-14-oxo-1(10),4,11(13)-germacratrien-12,6-olide, *Lachnospiraceae_UCG-002* enriching in Group HFD was significantly negatively correlated to PC(16 : 0/20 : 5(5Z,8Z,11Z,14Z,17Z)) and 6,7-Dihydro-4-(hydroxymethyl)-2-(p-hydroxyphenethyl)-7-methyl-5H-2-pyrindinium (*p* < 0.05). Additionally, *Eubacterium_xylanophilum_group* enriching in Group JPTGY was significantly positively correlated to cannabidiol dimethyl ether, 6,7-dihydro-4-(hydroxymethyl)-2-(p-hydroxyphenethyl)-7-methyl-5H-2-pyridinium, vinaginsenoside R14, 3-oxo-5*β*-chola-8(14), 11-dien-24-oic acid, C17 sphingosine-1-phosphocholine, erythromycin ethylsuccinate, 3-mercaptohexyl hexanoate, and N-(p-hydroxyphenethyl)actinidine (*p* < 0.05).

What is more, the metabolites of the Group JPTGY were inputted into MetaboAnalyst 5.0 to explore the metabolic pathways of JPTGY in the treatment of obesity. The results showed that the Group JPTGY may play a role in the metabolism of linoleic acid (LA), alpha-linolenic acid (ALA), glycerophospholipid, arachidonic acid (AA), and pyrimidine (Figure 8(f)).

## 5. Discussion

Research on metabonomics and gut microbiota in obesity has become a hotspot [36]. This study linked of corpulency phenotypes with gut microbiota and fecal metabolins unveils the latent causal link of JPTGY in the treatment of hyperlipidemia and obesity. In this study, the effects of JPTGY on the metabolism of lipid in blood be confirmed through serum biochemical indicators. Hyperlipoidemia is one of the aberrant lipidemia illnesses of lipometabolism dysfunction, the raised LDL-C or diminished HDL-C contents are tightly related to heart and blood vessel illnesses [37], and serum TC and TG contents are pivotal for ameliorating hyperlipoidemia [38, 39]. Dyslipidemia could deteriorate the progression of corpulency syndrome by stimulating inflammatory cytokines, inducing IR, and damaging glucose metabolic process, and disorders of lipid metabolism are another prominent feature of obesity [40]. The results herein suggest that JPTFY therapy could modulate hyperlipoidemia in HFD-fed obese mice and inhibits cardiovascular complications to a certain degree.

Nevertheless, the accurate causal link of JPTGY against corpulency and associated hyperlipoidemia is still elusive and requires more pieces of research. The intestinal flora is a key factor involving lipid metabolism and obesity [41], and changes in its components are related to aberrant inflammation and metabolisms like inflammation-related bowel illness, irritable bowel syndrome, and corpulency [42]. In recent years, it has become a new hotspot to analyze diseases by establishing an internetwork model of microbiota and metabolites [43]. In our study, the 16S rDNA analysis showed that the high-fat diet and JPTGY evidently affected the composition architectures of the intestinal flora in mice. To identify specific flora associated with HFD and JPTGY, we assessed the relative richness of intestinal flora at phylum levels.

At the phylum level, *Bacteroidetes* and *Firmicutes* were the 2 predominant phyla in the intestinal tract. *Bacteroidetes* had the potential to inhibit fat deposition in obese mice [44], *Firmicutes* were associated with the accumulation of lipid droplets, and their increased abundance could promote the absorption of fatty acids at the beginning of obesity [45]. Both of them were vital for modulating carbohydrate and lipometabolism of the host [46]. In the current study, the gut of HFD animals was featured by elevated richness of *Firmicutes*, diminished richness of *Bacteroidetes*, along with elevated ratio of F/B compared with Group NC, which coincided with the outcomes of “obesity flora” reported by Zhao et al. [47]. The human gut microbiota contained a small amount of *Proteobacteria*, and an increased abundance of *proteobacteria* was a sign of dysbiosis and a potential key to disease diagnosis [48]. *Proteobacteria* was considered to be one of the best sources of lipopolysaccharides (LPS), and the unstable intestinal microbial community characterized by abundant *proteobacteria* could induce obesity, metabolic disorders, and intestinal inflammation [48, 49]. In our study, a greater abundance of *Proteobacteria* was detected in the HFD mice and JPTGY decreased the level of this bacterium. The outcomes of the present research revealed that JPTGY could decrease the richness of *Proteobacteria*; hence, it might facilitate the reduction of metabolic disorders and intestinal inflammation initiated by HFD.

The LEfSe analysis noted that *Lachnospiraceae NK4A136 group* was one of the characteristic bacteria in the JPTGY group. Previous pieces of research reported that the elevated richness of *Lachnospiraceae NK4A136 group* facilitated the alleviation of aberrant metabolism, IR, and corpulency in HFD mice [50–52]. It was discovered that the richness of *Lachnospiraceae NK4A136 group* was related to inflammation in a negative manner [53]. Herein, our team discovered that JPTGY enriches the richness of *Oscillibacter* in mice as well. A study revealed that the relative richness of *Oscillibacter* was negatively related to inflammation, insulin resistance, and obesity-related indices in mice [9, 54]. Hence, our team speculated that how anticorpulency works of JPTGY might be owing to the elevated richness of *Lachnospiraceae NK4A136 group* and *Oscillibacter*. The enrichment of genera like *Lachnospiraceae NK4A136 group* and *Oscillibacter* in mice with JPTGY group indicated the role of JPTGY in obesity. The regulation of host lipometabolism and corpulency by intestinal flora relies on various intestinal flora metabolins [41]. SCFAs, like acetate, propionate, butyrate, isobutyrate, and isovalerate, were significant metabolins to microorganisms. It was discovered that SCFAs were vital for ameliorating energy metastatic process, glucose homeostasis, lipid metabolism, anti-inflammatory, enhancing the intestinal barrier, and modulating host immunity [55–57]. For example, butyrate and acetate can increase the energy consumption of human body, thus reducing body weight [58]. Previous studies indicated that supplementation with SCFAs effectively decreased the expressing level of peroxisome proliferator-activated receptor gamma (*PPARγ*) in mice, achieved the transformation from lipid synthesis to lipid oxidation, and alleviated the metabolic disorders induced by HFD [59]. In addition, SCFAs activation of GPR43 inhibits insulin-mediated fat accumulation [60]. It is known that *Erysipelotrichaceae*, *Erysipelotrichia*, *Clostridiaceae 1*, *Clostridium sensu stricto 1,* and *Intestinimonas* were producers of SCFAs in the gut, including butyrate [52, 61–64]. In addition, Chen et al. findings revealed that a greater richness of the 2 butyrate-generating microbes, *Clostridium sensu stricto 1* and *Clostridiaceae 1*, were concerned with lowering the incidence of T2D [64]. Changes in intestinal flora caused by HFD could lead to elevated intestine permeability, destruction of the intestinal barrier, high concentration of LPS, and metabolic endotoxemia. The combination of elevated LPS with toll-like receptor 4 (TLR4) could further induce fat inflammation and abnormal lipid accumulation in some tissues, causing metabolism illnesses like corpulency, IR, and MS [65–68]. As a directly targeted molecule for lipid transport and storage in adipose tissue, LPS participates in the progression of obesity and is a major inflammation factor leading to obesity [67, 69]. Chronic injection of LPS in mice leads to mild obesity [70]. *Turicibacter* was negatively correlated with LPS [71], which was beneficial to reduce intestinal inflammation. Apart from that, the predominant microbes in JPTGY mice also involved the genera of *Erysipelotrichales*, and *Parvibacter*, whereas those genera's effects on our health are still elusive. In the present study, JPTGY treatment could elevate SCFA-generating microbes and reduce LPS-generating microbes. These findings suggest that JPTGY may exert a favorable influence on the body via modulating the metabolites of the gut microbiota. Unfortunately, stool or circulation SCFAs and LPS contents were not identified herein, so the role of SCFAs and LPS in the identified correlation could not be verified. Future studies ought to corroborate the assumption of SCFA-generating microbes and LPS-generating microbes that influence lipometabolism and obesity risk through the generation of SCFAs and LPS. The accurate causal link by which JPTGY modulated the constituents and metabolins of intestinal flora requires more exploration in the future.

The gut microbiota regulated by JPTGY is mostly related to metabolic diseases, endocrine disease, and the terms of metabolic pathways showed changes in various lipometabolism, energy metabolic process, carbohydrate metabolic process, and amino acid metabolic process, which can offer enlightenment for the underlying causal links beneath the mitigation efficacy of JPTGY for the lipidic dysbiosis in rats caused by HFD. In the future, our team will utilize metagenomics sequence identification techniques to unveil the constituents and functions of gut flora at the microbe species level.

Gut microbiota affects host metabolism through a series of physiological, and the changes of metabolites also reflect the alternation of intestinal microbiota [72]. The volcano plot analysis clearly showed that HFD mice and JPTGY mice displayed a differentiation in feces metabolins vs. NC mice. In the present study, to determine groups of metabolins related to a special set of microbe genera, our team performed Pearson correlation analysis between the enriched genera and the feces metabolins. As presented in Figure 7, those associated metabolins could be classed into fatty acyls, indoles, sphingolipids, stilbenes, phenols, and others. In our study, 14 pivotal feces metabolins in response to JPTGY therapy were determined. Pearson correlation analysis revealed that those metabolitesare tightly associated with JPTGY effective genera of *Lachnospiraceae NK4A136 group*, *Oscillibacter*, *Turicibacter*, *Clostridium sensu stricto 1*, and *Intestinimonas*. In addition, metabolism pathway enrichment analyses revealed that LA metabolism path, ALA metabolism path, glycerophospholipid metabolism path, AA metabolism path, and pyrimidine metabolism path are latent target metabolism paths for JPTGY intervention (Figure 8(f)). LA and ALA are PUFAs and related to remarkably lower risks of diabetic diseases [73]. Bao et al. discovered that LA was lower in the serum of HFD-induced obese mice compared with normal mice [74]. Zhuang et al. reported that long-term intake of linolenic acid and alpha-linolenic acid could ameliorate adipose inflammation and IR for obese/overweight subjects via gut-adipose axis and sex-specific gut microbiota modulation, and alpha-linolenic acid may ameliorate glycolipid homeostasis [75]. The perturbation of membrane glyceryl phosphatide metabolic process will affect insulin excretion, influencing carbohydrate and lipid metabolism [76]. Disorders of glyceryl phosphatide metabolic process, ALA metabolic process, and LA metabolic process were associated with corpulency and corpulency-related illnesses [74]. Combined with metabolomics analysis, the metabolism of LA, ALA, glycerophospholipid, AA, and pyrimidine may be the significant pathway of JPTGY in the treatment of obesity. These results illustrated that the latent markers related to intestinal flora offered helpful data to better reveal the role of JPTGY in corpulency, and reinforced the treatment significance of JPTGY for corpulency. Those discoveries generally facilitate the understanding of the intricate interactions between obesity and the gut microbial ecosystem.

## 6. Conclusion

In summary, JPTGY is valid in mitigating HFD-triggered corpulency through regulating host lipometabolism, intestinal flora, and host metabolism. After JPTGY supplementation, the disorders in the metabolism of lipids were significantly weakened. In addition, JPTGY could adjust the structure, composition, abundance, and function of the gut microbiome of obese mice. Combined with metabolomics analysis, the metabolism of LA, ALA, glycerophospholipid, AA, and pyrimidine may be the significant pathway of JPTGY in the treatment of obesity. This study provides a new perspective for JPTGY to improve obesity through intestinal microbiota and metabolomics studies and further clarifies the mechanism of JPTGY in obesity treatment.

## Figures and Tables

**Figure 1:** Effects of High-fat diet and JPTGY on serum lipid profile. (a) TC; (b) TG; (c) LDL-C; and (d) HDL-C. Data were displayed as average ± SD (*n* = 10) and studied via one-way ANOVA ( ^*∗*^*p* < 0.05,  ^*∗*^ ^*∗*^*p* < 0.01 and  ^*∗*^ ^*∗*^ ^*∗*^*p* < 0.001).

**Figure 2:** Rarefaction curve and Shannon index analysis of the bacterial community in different treatments. The curves of every group tend to be flat with the increase of extracted sequence number, revealing that the sequence identification data amount of samples is acceptable, and more data amount will merely generate a little novel OTU.

**Figure 3:** The bacterial alpha diversity index in each group. (a) richness; (b) Shannon diversity; (c) Chao1 index; and (d) Phylogenetic diversity. The letters denote if there are remarkable diversities amongst the three treatments at *p* < 0.05. The identical letters denote no remarkable diversities and diverse letters, remarkable diversities. (e) Venn diagrams display core and shared intestinal flora species of the mice in diverse groups.

**Figure 4:** Bacterial community composition of three different treatments. (a) The *β*-diversity displaying as non-metric multi-dimensional scaling (NMDS) at the OTU level. (b) Hierarchical clustering analysis of UPGMA samples based on binary Jaccard distance.

**Figure 5:** Phylum composition of each treatment and the Firmicute/Bacteroidetes ratio in the phylum level. (a) The relative richness of the top 10 ranked phyla was displayed. (b) The ratio of F/B. The letters denote if there are remarkable diversities amongst the three treatments at *p* < 0.05. The identical letters denote no remarkable diversities and diverse letters denote remarkable diversities. Bar charts reflect the mean value and standard deviation for each group.

**Figure 6:** Representative microbes in different groups. (a) LDA scoring was calculated for taxa with differential richness in the feces flora of the Group NC, HFD, and JPTGY. The LDA scoring revealed the effect size and ranking of every differentially abundant taxon (LDA >3). (b) Cladogram reveals the phylogenesis distribution of function markers in response to JPTGY therapy. The area of the circle is associated with taxon richness in a positive manner.

**Figure 7:** Prediction of gut microbiota functional pathway in mice taking JPTGY. The heatmap showed distinguishingly expressed potential functions.

**Figure 8:** Metabolomics analysis among three groups. (a) The PLS-DA score plot; (b) volcano map of “HFD vs. JPTGY”; (c) volcano map of “HFD vs. NC”; (d) volcano map of “JPTGY vs. NC”; and (e) Pearson correlative analyses between the intestinal flora phyla and varied feces metabolins. Positive and negative associations are presented as red and blue in the heatmap, separately. The metabolins in correspondence to the metabolism path are displayed on the right. (f) Metabolic pathway analysis of Group JPTGY.

## Data Availability

The data used to support the findings of this study are available from the corresponding author upon request.
